The article "MiR-153 regulates expression of hypoxia-inducible factor-1α in refractory epilepsy" was retracted in 2025. Reasons: concerns about the data; concerns about the authorship.

# MiR-153 regulates expression of hypoxia-inducible factor-1α in refractory epilepsy

**DOI:** 10.18632/oncotarget.24012

**Published:** 2018-01-05

**Authors:** Guo-Hua Gong, Feng-Mao An, Yu Wang, Ming Bian, Di Wang, Cheng-Xi Wei

**Affiliations:** ^1^ Medicinal Chemistry and Pharmacology Institute, Inner Mongolia University for the Nationalities, Tongliao, Inner Mongolia, P.R. China; ^2^ Inner Mongolia Key Laboratory of Mongolian Medicine Pharmacology for Cardio-Cerebral Vascular System, Tongliao, Inner Mongolia, P.R. China; ^3^ First Clinical Medical of Inner Mongolia University for Nationalities, Tongliao, Inner Mongolia, P.R. China

**Keywords:** epilepsy, mTLE, miR-153, HIF-1α, luciferase reporter assay

## Abstract

Mesial temporal lobe epilepsy (mTLE), the most common type of temporal lobe epilepsy (TLE), is particularly relevant due to its high frequency of therapeutic resistance of anti-epileptic therapies. MicroRNAs (miRNAs) have been shown to be dysregulated in epilepsy and neurodegenerative diseases, and we hypothesized that miRNAs could be involved in the pathogenesis of MTLE. The present study aimed to explore the expression and functions of miRNA-153 in mTLE. The expression levels of miRNA-153 in refractory TLE patients were evaluated. The bioinformatics analysis showed that the potential target genes of miR-153 were involved in biological processes, molecular functions, and cellular components. miRNA-153 is significantly dysregulated in temporal cortex and plasma of mTLE patients. We identify HIF-1α as a direct target of miRNA-153, and luciferase reporter assays demonstrated that miR-153 could regulate the HIF-1αexpression via 3'-UTR pairing. These data suggest that miR-153 might represent a useful biomarker and treatment target for patients with mTLE.

## INTRODUCTION

Temporal lobe epilepsy (TLE) is a common disabling neurological disorder characterized by spontaneous, recurrent seizures, and affected individuals often require lifelong medication [1, 2]. Currently, antiepileptic drugs (AEDs) merely provide symptomatic control of seizures, but a third of patients remain refractory to AEDs [3, 4]. As a consequence, it is necessary to develop effective therapies to improve drug resistance. Mesial temporal lobe epilepsy (mTLE), the most common type of TLE patients, featured by refractory seizures worsen with time, and often become resistant to AEDs [5]. The clinicopathological manifestations of MTLE appear to be largely related to lesions of the medial temporal lobe structures [6]. However, the molecular mechanisms underlying AEDs resistance remain largely unknown.

MicroRNAs (miRNAs) modulate gene expression transcriptionally or posttranscriptionally by mainly binding to the 3′ UTR of target genes involved in signaling pathways [7, 8]. Recently, miRNAs has strong effects in cell fate during epilepsy and development of AEDs resistance [9]. MiR-153 is a conserved miRNA located within the PTPRN2 gene locus, and candidate regulator of teratogenesis and neurobehavioral impairment [10-12]. Although miR-153 is implicated in various neurodegenerative disorders including TLE, but the actual underlying mechanisms of miR-153 for AEDs resistance in mTLE are yet to be elucidated.

The article "MiR-153 regulates expression of hypoxia-inducible factor-1α in refractory epilepsy" was retracted in 2025. Reasons: concerns about the data; concerns about the authorship.

## RESULTS

In order to investigate the role of miR-153 in mTLE, firstly the miR-153 expression in a set of 22 surgical mTLE cases and 20 controls were evaluated. Our data reveal that miR-153 is downregulated in mTLE as compared with controls (Figure 1A, *P* < 0.01). Furthermore, the qRT-PCR and western blot analysis showed that the expression levels of HIF-1α were significantly upregulated in temporal cortex of mTLE (*P* < 0.01, Figure 1B, Figure 2A). Pearson’s correlation test showed there is a negative correlation between HIF-1α and miR-153 (*P* < 0.01). Furthermore, miR-153 showed lower expression in plasma of mTLE (Figure 2B, *P* < 0. 01). We examined the relationship between miR-153 in plasma and the clinical features in patients with mTLE. Frequency (*P* = 0. 018) and Engel classification (*P* < 0. 01) were found to be significantly associated with expression level of miR- 153.

**Figure 1:** The relative expression of miR-153 and HIF-1α were determined by qRT-PCR in mTLE patients (**A**) miR-153 expression levels were significantly lower in temporal cortex of patients with mTLE when compared with controls; (**B**) HIF-1α mRNA expression levels were significantly higher in temporal cortex of patients with mTLE when compared with controls.

**Figure 2:** (**A**) HIF-1α protein expression levels were significantly higher in temporal cortex of patients with mTLE when compared with controls; (**B**) miR-153 expression levels were significantly lower in plasma of 22 surgical patients with mTLE patients as compared with controls.

To demonstrate this conclusions further, potential target genes for miR153 were therefore searched for using bioinformatics software. On the basis of miRNA target analysis, HIF- 1α is a potential target mRNA of miR-153 (Figure 3A). Then, we co-transfected a firefly luciferase reporter vector containing the the WT or MUT 3′UTR of HIF-1α into HEK293 cells. Significantly, coexpression of miR-153 substantially repressed activity of the reporter that carried the wild-type but not mutant 3′UTR of HIF-1α (Figure 3B).

**Figure 3:** (**A**) HIF-1α is one of the candidates because miR-153 includes its potential binding sequences of the HIF-1αmRNA 3′-UTR; (**B**) Relative luciferase activity in HEK293 cells co-transfected with pGL3-HIF-1α-3′-UTRWT/MUT and miR-153 mimics or miRNA scramble control (miRcon).

The article "MiR-153 regulates expression of hypoxia-inducible factor-1α in refractory epilepsy" was retracted in 2025. Reasons: concerns about the data; concerns about the authorship.

To further confirm the regulatory effect of miR-153 on HIF-1α expression, we determined the changes of HIF-1α expression in pharmacoresistant astrocytes cells transfected with exogenous human miR-153 (miR-153 mimics) or suppressing miR-153 (miR-153 inhibitors). As expected, overexpression of miR-153 inhibited HIF-1α compared with mock or control transfections. In addition, inhibition of miR-153 could increase HIF-1α expression in astrocytes (Figure 4A and 4B).

**Figure 4:** (**A**) The relative levels of HIF-1α mRNA in astrocytes cells transfected with miR-153 mimics, miRNA mimic negative control (miR-con), miR-153 inhibitors (anti-miR-153), or miRNA inhibitor negative control (anti-miR-con). (**B**) The relative levels of HIF-1α protein in astrocytes cells transfected with miR-153 mimics, miRNA mimic negative control (miR-con), miR-153 inhibitors (anti-miR-153), or miRNA inhibitor negative control (anti-miR-con).

## DISCUSSION

Resistance to multiple AEDs have become increasingly attractive in refractory epilepsy therapy [14]. HIF-1α involved in various pathologic conditions, ranging from neurodegeneration to diabetes, and also MDR1 expression which correlated with epilepsy multidrug resistance [15].

MicroRNAs (miRs) are a group of small noncoding RNAs of about 22 nucleotides in length that negatively regulate specific gene expression, primarily through interaction with the 3′UTR of target mRNAs [16]. A growing number of specific miRNAs have definitely been reported in association with various types of epilepsy, including mTLE [17]. Multiple miRNAs have been identified to be responsible for seizure-related phases of TLE patients [18]. Although recent studies indicate the importance of miRNAs in TLE progression, its roles in mTLE still remain to be investigated.

In present study, our experiments showed that miR-153 regulated refractory epilepsy progression by regulating HIF-1α expression. We recognized that miR-153 is significantly decreased in plasma of patients with mTLE and the temporal cortex tissues. Bioinformatics approaches identified HIF-1α as a candidate miR-153 target gene. The results were confirmed by luciferase assay and the negative regulation of HIF-1α by miR-153 through at least one discrete 3′-UTR MRE. Mounting evidences confirmed the role of HIF1α in many biological processes such as the glycolytic pathway, angiogenesis, pH regulation, and pharmacoresistant epilepsy.

The expressions of HIF-1α mRNA and protein were both upregulated in in temporal cortex of patients with mTLE, which was in accordance with the results of a previous study. Consequently, we confirmed that HIF-1α is a direct target gene of miR-153 using luciferase assay. We showed a significant inverse correlation between the levels of HIF-1α and miR-153. miR-153 significantly inhibited the HIF-1α expression, however, inhibitiorof miR-153 could upregulated the HIF-1α levels.

The article "MiR-153 regulates expression of hypoxia-inducible factor-1α in refractory epilepsy" was retracted in 2025. Reasons: concerns about the data; concerns about the authorship.

Collectively, our study demonstrated that miR-153 is an important modifier of refractory epilepsy which regulates the expression of HIF-1α that contribute to pathogenesis of pharmacoresistant epilepsy. The present research suggest that miR-153 may serve as potential biomarkers of refractory epilepsy.

## MATERIALS AND METHODS

### mTLE patients and control group

Surgical specimens were obtained from 22 patients with mTLE who were undergoing anterior temporal lobectomy in our hospital with typical imaging features and pathologic confirmation. In addition, 20 patients who had undergone surgical treatment for head trauma or cerebral hemorrhage were also included. The study was approved by the University General Hospital. All human subject research was performed in accordance with institutional, national, and Declaration of Helsinki requirements, and before analysis, written informed consent was obtained from all patients.

### Brain tissue collection and RNA extraction

Temporal cortex tissues resected from 22 patients with refractory mTLE who had undergone anterior temporal lobectomy were collected. The 20 control samples of temporal neocortical tissues without abnormal pathological changes were obtained. None of patients in control group was ever diagnosed of epilepsy or seizures. Resected brain tissues were immediately frozen in liquid nitrogen for further studies.

For miRNA expression analysis, small RNAs from temporal cortex tissue from patients or controls were isolated using miRNA extraction kit (Qiagen) according to manufacture’s instruction. For detection of HIF-1α mRNA in brain tissue, RNA was extracted according to Trizol method (Invitrogen, USA).

### Plasma collection and RNA Extraction

5 ml blood samples from all mTLE cases, surgical control cases and healthy controls were collected in EDTA-containing tubes. Whole-blood samples were centrifuged at 1800 g for 20 min at 4°C after blood collection, and the upper plasma phase was carefully transferred into microcentrifuge tube. A second centrifugation at 1600 g for 10 min at 4°C to remove additional cellular debris and minimize contamination of cell-free nucleic acids derived from damaged blood cells. For long storage, plasma frozen in aliquots was kept at − 80°C until further analysis. Total RNA was extracted from 100 μ l of plasma samples using TRIzol LS reagent (Life Technologies) according to manufacturer’s instructions.

The article "MiR-153 regulates expression of hypoxia-inducible factor-1α in refractory epilepsy" was retracted in 2025. Reasons: concerns about the data; concerns about the authorship.

### Quantitative PCR (RT-qPCR)

For miRNA expression reverse transcription (RT) was carried out with the Universal cDNA Synthesis kit from Exiqon using 20 ng of total RNA. qPCR was performed using the ExiLENT SYBR Green master mix and miRCURY LNA Universal RT microRNA PCR primer sets following manufacturer’s recommendations (Exiqon INC., USA).

For target gene expression analysis cDNA synthesis was performed with High Capacity cDNA RT Kit (Life Technologies) and inventoried TaqMan Gene expression assays were used for qPCR together with TaqMan GenEx Master Mix (Life Technologies) following manufacturer’s instructions. The stably expressed human GAPDH gene was identified using the geNorm + module in qbase + and used as reference genes for normalization. Normalized relative expression levels for miRNA and mRNA were calculated using the qbase + software (Biogazelle NV, Zwijnaarde, Belgium).

### Western blot analysis

Lysate protein from tissue or cells was assayed by BCA (Pierce), and equal amounts of lysate protein (1–5 g) were loaded on to BisTris XT denaturing 10% polyacrylamide gels containing SDS (Bio–Rad Laboratories). Proteins were resolved by SDS/PAGE and transferred on to PVDF membranes. The samples were blocked and then incubated with the primary antibody diluted at 1:1,000 (mouse anti-HIF-1a monoclonal antibody, Novus, USA) at 4 C overnight. The membranes were washed and then incubated with HRP-labeled goat anti-mouse secondary antibody (1:10,000, Pierce, USA) at room temperature for 1 h, separately. The bands were detected using a chemiluminescent substrate (Millipore, USA). The GAPDH was used as an internal control. Gray values were measured using ImageJ Analysis Software (NIH). The relative expressions of samples in different duplications were standardized by a same sample of control group.

### Pharmacoresistant astrocyte model establishment and primary astrocyte cell culture

Pharmacoresistant astrocyte model was built using mechanical method modified from previous study [13]. Rat astrocytes were isolated and identified by immunocytochemical staining with GFAP. After 12 days induction, rat astrocytes grown under these conditions had high P-gp over-expression and optimal cell morphology were used in subsequent experiments.

### Transfection

MiR-153 mimics, miRNA mimic negative control (miRcon), miR-153 inhibitors (anti-miR-153), and miRNA inhibitor negative control (anti-miR-con) were purchased from GenePharma (Shanghai, China). Synthetic miR-153 mimics, miR-con, miR-153 inhibitors, and anti-miR-con were transfected into cells using Lipofectamine 2000 (Invitrogen) according to the manufacturer’s instructions.

The article "MiR-153 regulates expression of hypoxia-inducible factor-1α in refractory epilepsy" was retracted in 2025. Reasons: concerns about the data; concerns about the authorship.

### Luciferase reporting assay

The 3′ UTR of HIF-1α and the CMV promoter were amplified from human chromosomal DNA and pcDNA3.1 (+) and cloned into the pGL3-luciferase basic vector (Promega, Madison, WI, USA). Sequences of primers and cloning strategy are available on request. For the luciferase assays, 50 nM of miR-153 mimics or scrambled RNA were co-transfected with the reporter vector and the Renilla control vector (Promega, Madison, WI, USA) into the HEK293 cells by Lipofectamine 2000 (Invitrogen, Carlsbad, CA, USA). 24 h post transfection, the measurements were performed using the Dual luciferase re-porter assay kit (Promega, Madison, WI, USA). The HEK293 cells post the transfection for 24 h was lyzed for western blot analysis.

### Statistical analysis

All data were normally distributed and presented as mean values ± s.e. or s.d. as specified. Statistical differences between two groups were evaluated by two tailed unpaired Student’s *t*-test or with a two-sided Mann Whitney test with t approximation. In the case of multiple mean comparisons one-way analysis of variance (ANOVA) was used (Gnumeric 1.12.12; SPSS Statistics 19, IBM, USA). *P*-values < 0.05 were regarded as significant.
